# Application of 4% chlorhexidine to the umbilical cord stump of newborn infants in lower income countries: a systematic review and meta-analysis

**DOI:** 10.1186/s40748-019-0111-y

**Published:** 2019-10-17

**Authors:** Aklilu Abrham Roba, Maleda Tefera, Teshager Worku, Tamirat Tesfaye Dasa, Abiy Seifu Estifanos, Nega Assefa

**Affiliations:** 1 College of Health and Medical Sciences, Haramaya University, Harar, Ethiopia; 2 Department of Reproductive Health and Health Service Management, School Of Public Health, Addis Ababa University, Addis Ababa, Ethiopia

**Keywords:** Chlorhexidine, Umbilical cord, Cord separation time, Omphalitis, Neonatal mortality, Newborn infants, Low-income countries, Lower-middle income countries

## Abstract

**Abstract:**

There are conflicting results from large randomized controlled trials in different populations regarding the effectiveness of topical application of 4% chlorhexidine to the umbilical stump of newborn infants at reducing neonatal mortality. Meta-analysis and systematic review of trials performed in South Asia and Europe support 4% chlorhexidine application to reduce neonatal mortality, whereas trials performed in Sub-Saharan Africa do not. The aim of this review is to determine the effectiveness of 4% chlorhexidine application to the umbilical stump of newborn infants born in lower income countries in order to reduce neonatal mortality when compared with usual cord care.

Our search strategy included randomized trials published between January1^st^ 2000 and September 4th, 2018, that compared 4% chlorhexidine with usual cord care (“dry cord care”). The outcome variable of interest was neonatal mortality. Pooled relative risks (RR) with 95% confidence intervals (CIs) using a random-effects model were calculated. Nine trials were included, from six countries: Zambia, Tanzania, Bangladesh, Nepal, India and Pakistan, with a total of 257,153 participants. Five studies (*N* = 119,833) reported neonatal mortality. There was a 21% reduction in neonatal mortality among with 4% chlorhexidine application: pooled RR (95% CI) 0.79 (0.69–0.90), *P* = 0.0005. The incidence of omphalitis was decreased by 35% with 4% chlorhexidine (6 studies, *N* = 108,263): pooled RR (95% CI) 0.65 (0.56–0.75), *P* = 0.00001. Chlorhexidine application delayed the umbilical cord separation time (4 studies, *N* = 28,917): mean difference (95% CI) 2.71 (2.63–2.78) days.

In conclusion, this systematic review found that topical application of 4% chlorhexidine to the umbilical cord stump of newborn infants in lower income countries significantly reduces the incidence of neonatal mortality. Chlorhexidine also reduces the incidence of omphalitis, but prolongs umbilical cord separation time.

**Trial registration:**

Systematic Review Registration: CRD42018109280.

## Introduction

The first 4 weeks after birth are critical for the survival of newborn infants. Worldwide, 2.6 million neonatal deaths were estimated to occur in 2016, which translates to approximately 7000 deaths every day [1]. Omphalitis (infection of the umbilical cord) is an important cause of illness and death in newborn infants in developing countries [2]. Harmful traditional practices during cord cutting or tying, and the application of different substances to the fresh umbilical wound, may contribute to the entrance of infectious micro-organisms [3].

Chlorhexidine digluconate is a broad-spectrum antiseptic agent that is effective against a wide range of perinatal infectious microbials, as it strongly binds with their cell wall and disrupts their osmotic equilibrium [4]. It has been widely used for hand washing, oral care and medical purposes for decades, including for cleansing the umbilical cord and vaginal canal [5]. Because of its safety, efficacy, and low cost, chlorhexidine has been extensively evaluated as a means of preventing vertically acquired (intrapartum) neonatal infection.

A Cochrane review found that 4% chlorhexidine is effective to reduce neonatal mortality in settings with a high neonatal mortality rate (NMR) > 30/1000 live-births [6]. However, data is lacking on the effectiveness of chlorhexidine in a setting where the NMR is < 30/1000 live-births as well as for in-hospital deliveries [7, 8]. Globally, there are two important questions: 1) do the beneficial effects of chlorhexidine application warrant a change in the current recommendation of “dry cord care” (without chlorhexidine) in newborn infants [9]?, and 2) is the application of chlorhexidine as effective in the hospital setting as it is in the community setting?. Three trials from South Asia (Nepal [10], Bangladesh [11] and Pakistan [12]) found a reduction in neonatal mortality, while studies from Sub-Saharan Africa (Zambia [13] and Tanzania [14]) did not. No hospital-based studies have reported neonatal mortality [6].

Equipment used for umbilical cord tying or cutting may be a source of cord infection in newborn infants. One qualitative study in a rural community in Ethiopia found that umbilical cords were being cut with a razor, old blade, or even with a knife that was also used for cutting foodstuffs [3]*. C*ords were tied with a sewing thread, the thread from kerosene stoves, sisal thread, or thread or strips of cloth from a local blanket, traditional shawl or bed sheets. Butter, petroleum jelly and hair lotion were being applied to the cord [3]. Cord infections are associated with an increased risk of sepsis and neonatal mortality [15]. Therefore, in settings where exposure of the umbilical cord to potentially invasive pathogens is high, interventions that promote hygienic practices and topical cord antisepsis are recommended [16].

The aim of this systematic review and meta-analysis is to determine the effect on neonatal mortality of 4% chlorhexidine application to the umbilical stump of newborn infants, compared with “dry cord care”, in lower income countries. Omphalitis and cord separation time are secondary outcomes of interest.

## Methods

This Systematic review and meta-analysis was registered in PROSPERO with registration number CRD42018109280.

### Information sources and searching strategies

The following databases were searched from January1^st^ 2000 and September 4th, 2018: MEDLINE, PubMed, EMBASE, CINAHL, Web of Science direct (web of science core collection), Scopus, and Cochrane Central Register of Controlled Trials. In addition, we performed a manual search to retrieve unpublished studies and grey literature via Google Scholar and other sources. We used MeSH terms and search terms to construct a search string for each database that included terms ‘chlorhexidine’, ‘neonate’, and ‘umbilical cord’. For example, the following search strategy was used on PubMed: (“chlorhexidine gluconate”[Supplementary Concept] OR “chlorhexidine”[Mesh]) AND “infant, newborn”[Mesh]) AND “umbilical cord”[Mesh] AND ((clinical trial [ptyp] OR controlled clinical trial [ptyp] OR randomized controlled trial [ptyp]) AND “humans”[MeSH Terms]). To identify ongoing trials, we searched WHO trial registries in all three continents. Latin America and the Caribbean region were assessed through VHL regional portal using filtering (tw:((tw:(tw:((tw:(chlorhexidine)) AND (tw:(umbilical cord)) AND (tw:(newborn))) AND (instance:"regional”)))) AND (instance:"regional”) AND (collection:(“06-national”) AND db:(“IBECS” OR “LILACS”) AND mj:(“umbilical cord” OR “chlorhexidine” OR “bacterial infections” OR “umbilicus”))). After the searches, duplicate studies were removed, and remaining studies were screened for inclusion using the title and abstract. Included studies were then reviewed in full by two authors. Any differences in evaluation of studies were resolved by consensus of all authors. The PRISMA flow diagram [17] is shown in Fig. 1 and a summary of included studies in Table 1.

**Fig. 1:** Flow diagram showing literature search

**Table 1:** Summary table of trials

Study	Design and Sample size	Interventions	Comparator	Primary outcome/Other outcomes
Jamil,2018/Pakistan [20], Trial registration: Not found	Hospital-based RCT. I = 50 C = 50 T = 100	Chlorhexidine (liquid or gel form) were applied once daily for 7 days or till umbilical cord falls off.	Dry cord care	Presence of omphalitis was recorded as 38% in Dry care and 10% in the chlorhexidine group (*p* = 0.001)
Lyngdoh, D [18], 2018/ India, Trial registration: CTRI/2017/07/009146.	Hospital-based trial I = 35 (Chlorhexidine) C = 35 (Dry cord care) T = 105	He used chlorhexidine 4% as well as human breast milk in intervention arm	Dry cord care	4% chlorhexidine is very effective in reducing pathogenic bacteria colonization of the cord
Semrau, 2016/Zambia [13], Trial registration: NCT01241318	Cluster RCT. I^a^=18,450 C^b^=19,308 T^c^=37,758	Topical application of 4% chlorhexidine once per day until 3 days after cord drop.	Clean dry cord care	NMR^d^: 15·2/1000 live birth in IG^e^ NMR: 13·6/1000 live births CG^f^
Sazawal, 2016/Tanzania [14], Trial registration: NCT01528852	Community-based RCT. I = 18,015 C = 18,896 T = 36,911	4% chlorhexidine solution to the cord every day until 3 days after the cord had dropped off.	Dry cord care	NMR: 10.5/1000 live birth in IG NMR: 11.7/1000 live births CG
Khairuzzaman, 2015/ Bangladesh [21], Trial registration: Not found	Hospital-based RCT. I = 170 C = 170 T = 340	4% chlorhexidine solution	Dry cord care	The mean cord separation time in newborns of IG was significantly longer than CG (7.44 ± 3.75 Vs 4.83 ± 2.05 *p* < 0.001).
Mullany, 2013/Bangladesh [19], Trial registration: NCT00434408	Cluster-RCT I = 17,757 C = 9624 T = 27,381	Three arms IG: 1)4% chlorhexidine, 2) cleansing with soap and water	Dry cord care.	Cord separation time 1) Single group: 6.9 ± 2.87 days, 2) Multiple groups: 7.49 ± 3.08 days 3) Dry care: 4.78 ± 1.82 days
Sofi S, 2012/Pakistan [12]; Trial registration: NCT00682006	2X2 factorial, cluster-RCT. I = 4867 C = 4874 T = 9741	Four arms 1)4% chlorhexidine solution once daily up to 14 days along with soap and educational messages promoting hand washing. 2) The chlorhexidine solution only and 3) Hand washing only.	Dry cord care	A reduction in NMR (RR = 0·62, 95% CI 0·45–0·85); risk of omphalitis (RR = 0·58, 95% CI 0·41–0·82; No effect of hand washing for both outcomes
Arifeen, 2012/Bangladesh [11], Trial registration: NCT00434408	Community-based RCT. I = 19,608 C = 9924 T = 29,532	Three arms: 1) Multiple 4% chlorhexidine cleansing 2) Single 4% chlorhexidine cleansing	Dry cord care	NMR = 22·5 per 1000 LB in single chlorhexidine group, 26·6 per 1000 LB among multiple chlorhexidine groups and 28·3 per 1000 LB in dry cord care group.
Mullany L, C,2006/Nepal &Bangladesh [10], Trial registration: NCT00109616	Cluster-RCT. I = 4924 C = 5082 T = 10,006	Three arms: 1)4% chlorhexidine, 2) cleansing with soap and water	Dry cord care.	Neonatal mortality was 24% lower in the chlorhexidine group (RR = 0·76, [95% CI 0·55–1·04]) than in the DCC group Severe omphalitis in chlorhexidine clusters was reduced by 75% (incidence rate ratio 0·25, 95% CI 0·12–0·53.

^a^*I* Intervention

^b^*C* Control

^c^*T* Total

^d^*NMR* Neonatal Mortality Rate

^e^*IG* Intervention Group

^f^*CG* Control Group

### Eligibility criteria

We included RCTs that had been conducted in community or health facility settings, with individual or cluster randomization, and parallel or factorial designs. Studies that had been conducted in developing countries, and compared the effect of single or multiple topical applications of 4% chlorhexidine with “dry cord care” (applied nothing or soap and water only), irrespective of duration of follow-up in the neonatal period, were eligible. Studies that included all live births irrespective of gestational age or birth weight, had been published and were accessible before September 9th, 2018 and written in English were eligible. Studies that used other chlorhexidine strengths/concentrations, quasi-experimental studies, reviews, commentaries, editorials, and case series/reports were excluded.

### Description of the outcomes

The outcome variables of interest were neonatal mortality, defined as death within the first 28 days of life; omphalitis, defined as redness or swelling, with or without pus, in the skin surrounding the umbilical cord stump; and the time of umbilical cord separation, defined as the duration in days from birth to full separation of the umbilical cord from the stump.

### Risk of Bias

Two authors (AAR and TW) independently screened and evaluated studies using the Cochrane Risk of Bias Tool for Randomized Controlled Trials [22] (Table 2). Publication bias was explored using visual inspection of the funnel plot. Besides, Egger’s regression test [23] was carried out to check the symmetry of the funnel plot. Approximately symmetric funnel plots would indicate a “low risk” whereas asymmetric funnel plots would indicate a “high risk” of publication bias. Disagreements were resolved by consensus with other authors.

**Table 2:** Risk of bias of included studies

Author, year	Random sequence generation (selection bias)	Intention to treat (selection bias)	Blinding (performance bias)	Incomplete outcome data (attrition bias)	Selective reporting (reporting bias)	An overall decision on the quality of the study
Jamil,2018/Pakistan [20]	Moderate	unknown	unclear	High	unknown	Moderate risk of bias
Lyngdoh, D, 2018/ India [18]	Moderate	Moderate	unknown	Low	Low	Moderate risk of bias
Semrau, 2016/Zambia [13]	Low	Low	Unclear	Low	Low	Low risk of bias
Sazawal, 2016/Tanzania [14]	Low	Low	Not blind	Low	Low	Low risk of bias
Khairuzzaman, Md, 2015/ Bangladesh [21]	Unclear	Low	Unclear	Low	Low	Moderate risk of bias
Mullany, 2013/Bangladesh [19]	Low	Low	High	Low		Low risk of bias
Soofi S, 2012/Pakistan [12]	Low	Unclear	Low	Low	Low	Low risk of bias
Arifeen, 2012/Bangladesh [11]	Low	Low	Low	Low	Low	Low risk of bias
Mullany L, C,2006/Nepal &Bangladesh [10]	Low	Low	Low	Low	Low	Low risk of bias

### Statistical analysis

Data synthesis and statistical analysis were carried out by three authors (AAR, NA, and MT). Meta-analysis was conducted using Review Manager Version 5.3 software [24] for Relative Risk (RR) for neonatal mortality and omphalitis; mean difference (95% confidence interval [CI]) was used for cord separation time. Heterogeneity between studies was examined using the *I*^*2*^ statistic described by Higgins et al. [25] and *p*-value: *P* < 0.10 or *I*^*2*^ > 75% were considered as evidence of significant heterogeneity, which was explored further by sensitivity analysis. Sub-group analysis was conducted between Sub-Saharan and South Asian countries as well as studies of hospital and community settings.

## Results

### Study descriptions

A total of 12 RCTs were included in this systematic review and meta-analysis. The outcome of neonatal mortality was reported in five RCTs, conducted in Zambia, Tanzania, Bangladesh, Nepal and Pakistan with a total of 119,973 participants. Omphalitis was reported in six RCTs, conducted in Zambia, Tanzania, Bangladesh, Nepal and Pakistan with a total of 108,263 participants.

Four RCTs, from Bangladesh, India and Nepal with a total of 28,917 participants, reported cord separation time. Fig. 1.

### Neonatal mortality

The application of 4% chlorhexidine reduced the pooled incidence of neonatal mortality by 21% compared with dry cord care (Fig. 2): pooled RR 0.79; 95% CI: 0.69–0.90; *P* = 0.0004; random-effects model. There was minimal heterogeneity between trials for this outcome (I^2^ = 44%, χ^2^ = 7.11, *P* = 0.13).

**Fig. 2:** Effect of 4% chlorhexidine application on neonatal mortality

Of the five studies, four [10–14] were conducted in a community setting, while one was conducted in hospital neonatal intensive care unit [20]. Two studies were conducted in Sub-Saharan Africa of Zambia and Tanzania [13, 14], and three in South Asia, Nepal, Bangladesh and Pakistan [10–12]. All except the Zambian study [13, 26] were conducted in countries with a high NMR > 30/1000 live-births. All of the studies enrolled predominantly home delivered newborn infants. The Tanzanian study recruited participants from both the hospital and community (home based) setting, with more than half of the participants born in hospitals [14]. In the Zambian study [13], 11·4% of births in the chlorhexidine group and 16·1% of the dry cord care group were born in hospitals [13]. Sub-group analysis based on geography found that 4% chlorhexidine reduced neonatal mortality by 43% in South Asia (RR [95% CI] 0.57 [0.42–0.76]) and 30% in Sub-Saharan Africa (RR [95% CI] 0.70 [0.67–0.74]) (Fig. 2).

### Omphalitis

The application of 4% chlorhexidine reduced the pooled incidence of omphalitis by 35% compared with dry cord care (Fig. 3): pooled RR 0.65; 95% CI: 0.56–0.75; *P* = 0.00001; random-effects model. There was significant heterogeneity between studies for this outcome (I^2^ = 91% χ^2^ = 56.51, *P* = 0.00001).

**Fig. 3:** 4% chlorhexidine application on the incidence of omphalitis

Sub-group analyses of Sub-Saharan Africa versus South Asian settings (Fig. 4) and community versus hospital-based care (Fig. 5) were performed. In Sub-Saharan Africa, 4% chlorhexidine reduced the incidence of omphalitis by 30%: pooled RR (95% CI) 0.70 (0.67–0.740), I^2^ = 0, χ^2^ = 0.26, *P* = 0.00001. In the South Asian setting, there was a 43% reduction in omphalitis: pooled RR (95% CI) 0.57 (0.42–0.76), but there was substantial heterogeneity between studies (I^2^ = 94%, *P* = 0.00001) (Fig. 4).

**Fig. 4:** Sub-group analysis based on geography; 4% chlorhexidine application on the incidence of omphalitis

**Fig. 5:** Sub-group analysis based on setting; 4% chlorhexidine application on the incidence of omphalitis

Additional subgroup analysis found that 4% chlorhexidine reduces omphalitis in both the community setting (pooled RR 0.65 [0.55–0.76]) and hospital setting (pooled RR 0.49 [0.18–1.36]), but there was substantial heterogeneity between studies for both subgroup analyses (Fig. 5).

### Cord separation time

The application of 4% chlorhexidine increased the cord separation time by a mean difference (95% CI) 2.12 (0.95–3.29) days, I^2^ = 100%, *p* = 0.0004 (Fig. 6). Sub-group analyses of community versus hospital-based study (Fig. 7) were performed. 4% chlorhexidine increased cord separation time by a mean difference (95% CI) 2.52 (1.91–3.12) days, I^2^ = 0%, *p* = 0.00001 in hospital settings and (95% CI) 1.90 (0.30,4.49) days, I^2^ = 100%, *p* = 0.02 in community.

**Fig. 6:** 4% chlorhexidine application on time of cord separation

**Fig. 7:** 4 Sub-group analysis based on Geography; 4% chlorhexidine application on cord separation time

## Discussion

This review found that 4% chlorhexidine application to the umbilical stump of newborn infants in lower income countries significantly reduces neonatal mortality. Previously, individual studies from sub-Saharan Africa (Zambia and Tanzania [13, 14]) found that 4% chlorhexidine application to the umbilical cord did not reduce neonatal mortality, whereas studies from South Asian countries [10–12] found that it did. However, our pooled analysis found a 30% reduction of neonatal mortality in sub-Saharan Africa. In countries with high rates of home births, application of 4% chlorhexidine significantly reduces neonatal mortality. All except the Zambian study [13] were conducted in countries with a high rate of home births (> 40%). Bangladesh, Pakistan and Nepal have high home deliveries of 93, 80 and 58% respectively whereas Tanzania has 48%.

There has been debate as to whether to change the current WHO guideline that advocates dry cord care for newborn infants. In their correspondence, Osrin and Colbour argue that there is no need to change current dry cord care practice [22]. In contrast, Goldenberg and colleagues support the application of 4% chlorhexidine as they were convinced by its positive effect on the incidence of both neonatal mortality and omphalitis [23]. Based on Sankar’s review, the topical application of chlorhexidine was estimated to reduce neonatal mortality by about 15% and omphalitis by 30% (8) in infants born in settings that are comparable to those settings in our study. Sharif found a pooled reduction in neonatal mortality of 20% and in omphalitis by 60% [24].

An important consideration before the introduction of universal 4% chlorhexidine cord care in lower income countries is adverse effects of the therapy. Trials in Germany [27] and Pakistan [28] have shown chlorhexidine prevents skin erosion, irritation, omphalitis, erythema, umbilical granuloma, purulence, bleeding, discharge and weeping of the navel. Another trial in Pakistan showed there were no adverse effects [12], whereas there are case-reports of adverse effects in preterm and low birth weight infants [29–33]. Ultimately, the amount of exposure to chlorhexidine that can be considered safe is not known [34].

The strength of our current meta-analysis is that the studies included are RCTs from both community and hospital settings. It included seven large trials from two large continents: Asia and Africa. In general, the risk of bias of the studies was low (Table 2). However, there are some limitations of our results. Some of the studies included in the meta-analysis reported neonatal deaths from recruitment, whereas others excluded deaths on the day of life associated with birth asphyxia. Some of the studies were not blinded, especially those from community settings.

## Conclusion

Topical application of 4% chlorhexidine on the umbilical cord of newborn infants born in lower income countries reduces neonatal mortality by 21% and omphalitis by 35%. Chlorhexidine use delays cord separation time by about 2.5 days in the hospital setting and 2 days in the community. The intervention is effective in both community-based as well as health facility settings for the prevention of omphalitis. We recommend guidelines consider including 4% chlorhexidine application as routine practice in these settings.

## Data Availability

The data that support the review findings of this study are available upon submitting a reasonable request to the corresponding author.

## Abbreviations

AAR: Aklilu Abrham Roba
CI: Confidence Interval
LB: Live Birth
MeSH: Medical Search Heading
MT: Maleda Tefera
NA: Nega Assefa
NMR: Neonatal Mortality Rate
RCT: Randomized Controlled trial
RR: Risk Ratio
SSA: Sub-Saharan Africa
TTD: Tamirat Tesfaye Dasa
TW: Teshager Worku
